The article "Nonalcoholic fatty liver disease experiences accumulation of hepatic liquid crystal associated with increasing lipophagy" was published in 2020. Journal: Cell Biosci.

# Nonalcoholic fatty liver disease experiences accumulation of hepatic liquid crystal associated with increasing lipophagy

**DOI:** 10.1186/s13578-020-00414-2

**Published:** 2020-04-06

**Authors:** Liyang Wang, MengMeng Xu, Odell D. Jones, Zhongguang Li, Yu Liang, Qiuxia Yu, Jiali Li, Yajun Wu, Xinjuan Lei, Boling He, Huimin Yue, Liqin Xiao, Rong Zhou, Wei Zhang, Xin Zhou, Yuhui Zhang, Joseph L. Bryant, Jianjie Ma, Yingli Liu, Xuehong Xu

**Affiliations:** 1 Key Laboratory of the Ministry of Education for Medicinal Resources and Natural Pharmaceutical Chemistry, National Engineering Laboratory for Resource Development of Endangered Crude Drugs in Northwest of China, Xi’an, 710062 China; 2 Laboratory of Cell Biology, Genetics and Developmental Biology, Shaanxi Normal University College of Life Sciences, Xi’an, 710062 China; 3 Department of Pediatrics, Columbia University, New York, NY 10032 USA; 4 University of Pennsylvania School of Medicine ULAR, Philadelphia, PA 19144 USA; 5 Ohio State University School of Medicine, Columbus, OH 43210 USA; 6 University Hospital Shaanxi Normal University, Xi’an, 710062 China; 7 Institute of Basic and Translational Medicine, Xi’an Medical University, Xi’an, 710021 Shaanxi China; 8 University of Maryland School of Medicine, Baltimore, MD 21201 USA

**Keywords:** High-fat induced fatty liver disease, Non-alcoholic fatty liver disease (NAFLD), Liquid crystal, Phase transition, Biopsy diagnostics

## Abstract

**Background:**

In the past 30 years, incidences of non-alcoholic fatty liver disease (NAFLD) has risen by 30%. However, there is still no clear mechanism or accurate method of anticipating liver failure. Here we reveal the phase transitions of liquid crystalline qualities in hepatic lipid droplets (HLDs) as a novel method of anticipating prognosis.

**Methods:**

NAFLD was induced by feeding C57BL/6J mice on a high-fat (HiF) diet. These NAFLD livers were then evaluated under polarized microscopy, X-ray diffraction and small-angle scattering, lipid component chromatography analysis and protein expression analysis. Optically active HLDs from mouse model and patient samples were both then confirmed to have liquid crystal characteristics. Liver MAP1LC3A expression was then evaluated to determine the role of autophagy in liquid crystal HLD (LC-HLD) formation.

**Results:**

Unlike the normal diet cohort, HiF diet mice developed NAFLD livers containing HLDs exhibiting Maltese cross birefringence, phase transition, and fluidity signature to liquid crystals. These LC-HLDs transitioned to anisotropic crystal at 0 °C and remain crystalline. Temperature increase to 42 °C causes both liquid crystal and crystal HLDs to convert to isotropic droplet form. These isotropic HLDs successfully transition to anisotropic LC with fast temperature decrease and anisotropic crystal with slow temperature decrease. These findings were duplicated in patient liver. Patient LC-HLDs with no inner optical activity were discovered, hinting at lipid saturation as the mechanism through which HLD acquire LC characteristics. Downregulation of MAP1LC3A in conjunction with increased LC-HLD also implicated autophagy in NAFLD LC-HLD formation.

The article "Nonalcoholic fatty liver disease experiences accumulation of hepatic liquid crystal associated with increasing lipophagy" was published in 2020. Journal: Cell Biosci.

**Conclusions:**

Increasing concentrations of amphiphilic lipids in HLDs favors organization into alternating hydrophilic and hydrophobic layers, which present as LC-HLDs. Thus, evaluating the extent of liquid crystallization with phase transition in HLDs of NAFLD patients may reveal disease severity and predict impending liver damage.

## Background

Non-alcoholic fatty liver disease (NAFLD) is a disorder of excessive fat accumulation (steatosis) in the liver of those who consume little to no alcohol [1, 2]. With the increase of rich foods in the diets of Western counties and developing countries around the world, NAFLD has become a rising cause of hepatic steatosis since its first reported in 1983 [3–5]. Up to 25% of adults in the United States has NAFLD, with more than 80% of the obese population affected by the disease. Because there are often no initial symptoms for patients with NAFLD and the disease can only be treated by addressing the underlying condition, over time NAFLD patients often progress to severe liver fibrosis and cirrhosis [6, 7]. Because of this difficulty in treatment, liver disease is becoming one of the top leading causes of death in societies where rich diets are common. Liver disease is becoming an increasing problem in developing countries as well. According to the Asia–Pacific Working Party guidelines on NAFLD, over-nutrition has increased the prevalence of NAFLD in the Asia Pacific regions from 23.3 to 31.9% in the past 30 years [8]. Due to increasing childhood obesity, NAFLD has also become the primary form of liver disease in both children and adolescents [5, 9, 10].

Only a few genetic variations and environmental factors have been contributed to the development of the complex metabolic associated syndrome that is NAFLD. Two variants of the triacylglycerol lipase gene *PNPLA3* have been associated liver disease, one linked to severity of hepatic steatosis while the other affects hepatic triglyceride content by association with *TM6SF2*, a regulator of hepatic fat metabolism [11, 12]. Polymorphisms at *APOC3*, a gene controlling hepatic triglyceride content, have also been linked to NAFLD, but was later contradicted by a meta-analysis on *APOC3* polymorphisms and NAFLD risk [13, 14]. We have also previously reported a novel association of *NG37* with high fat diet induced NAFLD [15]. Our data demonstrated that overexpression of *NG37* in a transgenic mouse model results in liver enlargement and cardiac dysfunction in a high-fat diet dependent matter. This model provided a direct link between genetic predisposition and nutritional factors in hepatic lipid deposition [15].

The article "Nonalcoholic fatty liver disease experiences accumulation of hepatic liquid crystal associated with increasing lipophagy" was published in 2020. Journal: Cell Biosci.

Until now, the specific genetic causes of NAFLD were unclear, making it difficult to identify patients at high risk for severe NAFLD that is likely to progress to steatohepatitis, fibrosis, and cirrhosis. Recently, some researches have claimed that hepatic cholesterol crystals and crown-like structures distinguish Nonalcoholic steatohepatitis (NASH), an advanced subtype of NAFLD, from simple steatosis in humans [16]. These cholesterol crystal structures can also be detected in the fatty livers of thyroidectomized chickens and a murine NASH model [17, 18]. In our *NG37* murine model, we occasionally found lipid droplets (LD) as optically active anisotropic liquid crystals (LC) in the hepatocytes of NAFLD mice. These anisotropic liquid crystal hepatic lipid droplets (LC-HLD) can transform into isotropic LD under the right condition. Both these LC-HLDs and isotropic HLDs could also transition into crystal structures. Based on increasing investigations on unveiling molecular mechanism of diseases with phase transition and separation [19–21], it is certain that the liquid crystalline could be important clue of NAFLD genesis. This phenomenon of LC to crystal transition in vitro indicates that the buildup of lipids inside hepatocytes from overnutrition could be being stored as liquid crystals. Thus we hypothesized that the crystal and crown-like structures previously identified in human hepatocytes of NASH patients are likely the final form of LC-HLD after further over-accumulation of cholesterols [16, 17, 21].

## Materials and methods

### Human subjects and animals maintenance

All animal care and experiment procedures were conducted in accordance with protocol approved by the Animal Care and Use Committee of Shaanxi Normal University. All human studies were conducted according to the principles of the Declaration of Helsinki, and the study protocol were approved by the Institutional Ethics Committee of the Shaanxi Normal University with written informed consents from Alenabio (Xi’an, China). Tissues for detecting the phase characteristics of the tissues and the expression of the protein in autophagy pathway were collected from ten patients.

All C57BL/6J mice were housed in clean-normative animal rooms (temperature ~ 25 °C, ventilation, 12 h light/dark cycle) and bred under standard conditions. Male or female mice (n = 40, age: 5–8 weeks) were weighed and divided equally into two groups. The control group were fed with regular mouse chow (China National Standard GB14924.3-2010) purchased from animal core facility of Xi’an Jiaotong University School of Medicine Animals (Xi’an, China), and supplied with boiled tap water. The experiment group were supplied with high fat (HiF) diet produced in house as previously described, containing 88% standard diet, 10% lard and 2% cholesterol. The HiF diet group also received 0.2% more sucrose in water (w/v, changed daily) compared to the control group [22]. Both diets and water were provided on a free-taking principle. After 25 weeks, animals were euthanized by cervical dislocation prior to dissection for sample collection.

The article "Nonalcoholic fatty liver disease experiences accumulation of hepatic liquid crystal associated with increasing lipophagy" was published in 2020. Journal: Cell Biosci.

### Sample preparation and histological analysis

Fresh livers were dissected from mice and processed for paraffin section and cryo-section preparation. For paraffin section, samples were fixed by 4% neutral-buffered paraformaldehyde, dehydrated through gradient alcohol, cleared with xylene, embedded in paraffin and cut into 5–8 μm sections. For cryo-sectioning, the samples were placed into cryomatrix embedding agent (OTC), frozen without delay and cut at a thickness of 10 μm.

Paraffin and cryo-sections were then processed for histological analysis via Hematoxylin and Eosin (H&E) and Masson and Sirius red staining as previously described [23, 24]. Slides were rapidly dehydrated in gradient ethanol and cleared in xylene after staining before being permanently preserved in neutral balsam between glass cover slips.

### Polarization microscopy, phase transition and fluidity analysis

The samples obtained from hepatic lipid droplets of HiF diet induced NAFLD were prepared with both smear-slide and cryosectioned in media with 20% glycerol PBS. Optical activity was recorded under non-crossed polarizer and analyzer for conventional observations. Birefringence of specimens observed between two crossed prisms (or polarizer and analyzer) were documented for advance analysis as previously described [24–26].

Observation of optical activity proceeded with XS-213A-P Polarization Microscope (Jnoec Ltd, Jiangnan, Nanjing, China) and Zeiss Observer. A1 microscope affiliated with additional polarization accessory. A combination of inverted microscope PE120 peltier system (Linkam Scientific Instruments, UK) and XS-213A-P polarization microscope was carried out for our experiments. The PE120 peltier system was configured to run with a 5 mm aperture at a heating–cooling rate with a range of 0.1 to 20 °C/min. Temperature stability was set at 0.1 °C and controlled with the RS232 temperature controller. Temperatures of phase transition between anisotropic status and isotropic phases, including liquid crystal and crystal status, were recorded according to the observation of sample birefringence activities between polarizer and analyzer. Phase transition is define as a state transition between any two states among liquid state (optical isotropic with fidelity), crystal state (optical anisotropic without fidelity) and liquid–crystal state (optical anisotropic with fidelity). Two phases related to a transition are labelled as subscript of Ph and arrow in subscript indicates transition from first state to second state.

The article "Nonalcoholic fatty liver disease experiences accumulation of hepatic liquid crystal associated with increasing lipophagy" was published in 2020. Journal: Cell Biosci.

Pressure application-and-release experiments were utilized to characterize fluidity of birefringent hepatic lipid droplets obtained from HiF diet induced NAFLD mice. After samples were mounted between glass slides and over-slips with PBS-glycerol media, pressure was applied onto the glass cover-slip with a rubber applicator, and subsequently released. Images of the entire process were documented continuously under polarization microscope and further image analysis conducted on these records.

### X-ray diffraction analysis

For characterization of optical activity, NAFLD livers were directly applied on to the specimen plate and observed as previously described [15, 24]. The XRD (X-ray diffraction) patterns were obtained on the wide-angle goniometer of D/max-rA diffractometer in diffraction angle (2θ) of 5–45° with CuK α radiation, graphite monochromator, slit sizes of 1°(DivS)–10 mm(DivH)–1°(SctS)–0.3 mm(RecS), Scan 4.00, and power 40 kV × 100 mA. Samples of normal livers, HiF induced NAFLD livers and purified extracts from HiF induced NAFLD livers were measured at the above condition, which were clutched between two non-diffraction films to reduce movement and dehydration.

### Thin-layer chromatography

Thin-layer chromatography (TLC) was performed on a commercial made standard plate (QingDao Ocean Product, Ltd. Qingdao, China) coated with a thin layer of silica gel as the stationary phase. Fresh tissues were cut into small pieces and pulped in a double volume of 0.1 M phosphate buffer solution (pH 7.4). The up-suspended substances were then extracted by mixing with triple volume of chloroform/methanol (1/2, V/V), and centrifuged on 22.4*g* for 10–15 min followed by sample drying. The samples were then applied on the silica plate along with standard samples, including cholesterol, lecithin and cholesteryl oleate. A mix of chloroform–methanol–water (65:10:1) was used as the mobile phase and several locations within each samples was visualized under 254 nm UV light.

The article "Nonalcoholic fatty liver disease experiences accumulation of hepatic liquid crystal associated with increasing lipophagy" was published in 2020. Journal: Cell Biosci.

### Immunofluorescence analysis

Paraffin sections of HiF diet induced NAFLD tissues and cryo-sections of patient fatty liver tissue were processed for immunofluorescence staining. For paraffin embedded samples, antigens were retrieved in Target Retrieval Solution (DAKO North America, Inc., Carpinteria, CA, USA) and antigen of frozen samples were retrieved in methanol/acetone (V/V, 1/1). After these sections were blocked with 1% BSA, they were incubated with Anti-MAP1LC3A (1:50, Abcam, USA) and Anti-Beclin 1 (1:100, Abcam, USA). Secondary antibodies, Fluorescein (FITC) AffiniPure goat anti-mouse IgG (1:50, Jackson ImmunoResearch Lab, INC) and Rhodamine Red™-X (RRX) AffiniPure goat anti-rabbit IgG (1:50, Jackson ImmunoResearch Lab, INC., west Grove, PA, USA). Nuclei were counterstained by DAPI in these immune-stained sections. Immunofluorescence images were captured under confocal laser scanning microscopy (Olympus confocal microscope FV1200).

### Statistics

Conventional and polarized images of HLD were analyzed for birefringence intensity and quantified using the image analysis software ImageJ 1.50d (NIH, Bethesda, MD, USA). Statistical analyses were performed via SPSS 22 (IBM, Armonk, NYC) and charts compiled using GraphPad Prism 7.00 (GraphPad Software, La Jolla, CA).

## Results

### High-fat diet generates optical birefringent crystal structures in the liver of NAFLD animals

To generate NAFLD animals, litter mate C57BL/6J mice were fed with either a high-fat diet (HiF) or a normal diet as previously described [15, 22]. After 25 weeks of this diet, mice of both groups were euthanized and samples harvested. Both HiF diet and control diet livers were treated with the standard FEDXT procedure (the treatment combination of formaldehyde fixation, ethanol gradient dehydration, and xylene for transparent is short for FEDXT) prior to paraffin embedding and further histology and optical activity analysis. The standard cryo-sections procedures for histological and crystal analysis were also conducted on the livers as previously described [23–25]. To measure optical activity, sections were directly mounted with PBS and polarized microscopy performed without FEDXT treatment.

Conventional light microscopy was performed on paraffin-embedded sections and Cryo-sections of the HiF diet livers and normal diet controls. Histological staining with H&E, Sirius Red and Masson’s trichrome on paraffin-embedded sections confirmed the presence of lobular inflammation, steatosis, and light perisinusoidal fibrosis in HiF diet livers, while these pathologies were absent from non-HiF diet counterparts (Fig. 1A a–d). Cryo-section specimens stained with H&E, Sirius red, and Masson’s trichrome displayed results similar to paraffin-embedded sections, with inflammation, steatosis, and light perisinusoidal fibrosis in the HiF diet group only (Fig. 1B a–d). However, polarization microscopy revealed dramatic differences in optical activity between paraffin-embedded and cryo-section samples. There was no detectable birefringent activity in either the cryo-sectioned or paraffin embedded livers of normal diet mice (Fig. 1B e), while cryo-sections from hiF diet mice displayed optical birefringent activities in the form of needle and arch-shaped crystals (Fig. 1B f). Smear samples from normal diet and HiF diet mice confirmed the slide preparations findings (Fig. 1C). The birefringence of cryo-sections crystal and liquid crystal droplets are studied under differently angled polarized light to demonstrated their birefringence (Fig. 1D). There is a visible difference between paraffin embedded and cryo-preserved samples of HiF diet livers, with cryo-preserved samples retaining much of the optical activity.

The article "Nonalcoholic fatty liver disease experiences accumulation of hepatic liquid crystal associated with increasing lipophagy" was published in 2020. Journal: Cell Biosci.

**Fig. 1:** Conventional preparation effect on crystal optical activity of NAFLD hepatocytes. **A** The standard FEDXT procedure (formaldehyde fixation, ethanol dehydration, and xylene transparency) was used to prepare control and HiF diet induced NAFLD livers for H&E (Aa and Ab) and Masson Trichrome (Ac and Ad) histology, which showed control hepatocytes and hepatocytes with large empty vacuoles respectively. **B** H&E (Ba and Bb) and Masson Trichrome (Bc and Bd) staining of the same NAFLD and control samples prepared by cryo-section showed the same histology. Images of these specimens under polarized light prior to the staining process shows a lack of birefringence in the control group and birefringent crystals in NAFLD livers (Be and Bf). **C** Smear samples from control liver and NAFLD liver observed under polarized light showed the same non-birefringent and birefringent activity, respectively (Ca and Cb). **D** Cryo-sections of HiF diet induced NAFLD livers are shown after cryo-sectioning (Da) and post crystal-to-isotropic-droplet-to-liquid–crystal phase transitions (Db). Magnifications of these corresponding anisotropic crystals and anisotropic Maltese cross LC-HLD under polarizers are shown at a non-crossed angle of 45° (Dc and Dd) and crossed angle of 90° (De and Df)

The optical activity of hepatic crystal structures extracted from HiF fed NAFLD mouse livers were examined by XRD and found to diffract within the detection spectrum of 5° to 45° degrees (Fig. 2b). This XRD spectral peak pattern was comparable to the XRD pattern of unextracted, fresh HiF specimens (Fig. 2a) and normal liver controls have no diffraction (Fig. 2c). These peaks most closely identified with those of cholesteryl oleate (Fig. 2d), but less well with that of cholesterol and lecithin. The XRD spectrum of these extract specimens in its fully crystalline form identified diffractions at lattice planes d(Å) of 9.634, 5.899, 4.887, 4.563, 4.437 and 4.081 corresponding to I/I_0_ (17), I/I_0_ (24), I/I_0_ (100), I/I_0_ (54), I/I_0_ (15) and I/I_0_ (29) in the detection spectrum of 5° to 45°. Among all diffractions of the purified extracts from NAFLD livers, the most diffraction peaks match with that of cholesterol oleate listed in Table 1 except three lattice planes d(Å) of 9.634, 4.437 and 4.081 corresponding to I/I_0_ (17), I/I_0_ (15) and I/I_0_ (29) are unidentified crystalline form. All liver samples were stored at 4 °C and brought to room temperature prior to XRD examination. Thin-layer chromatography revealed that cholesterol oleate is the main component of HLD from HiF diet induced NAFLD livers, which support the above XRD data analysis (Fig. 3).

The article "Nonalcoholic fatty liver disease experiences accumulation of hepatic liquid crystal associated with increasing lipophagy" was published in 2020. Journal: Cell Biosci.

**Fig. 2:** Characterization of HiF diet induced NAFLD mouse liver and hepatocyte extracts. **a** Diffraction patterns of frozen NAFLD liver by XRD diffraction angle (2θ) of 5–45° and intensity (counts/second) had a set of diffraction peaks (**a**) matching the diffraction pattern of liver extracts (**b**), and were not observed in the controls (**c**). These diffraction peaks corresponds with the diffraction pattern of cholesteryl oleate (**d**)

**Table 1:** X-ray diffraction pattern of the crystal from HiF diet induced NAFLD liver and their purified extracts

Standard cholesteryl oleate		HiF diet induced NAFLD liver		Purified extracts from NAFLD liver	
d(Å)	I/I0	d(Å)	I/I0	d(Å)	I/I0
		9.6344	17	9.9273	21.7
9.3311	48.1			9.6349	12.6
9.3263	48.8			9.621	13.2
8.1815	3			8.4386	2.9
7.7929	11.6			7.9114	7
6.9783	2.7			7.0791	2.7
5.927	12.5	5.8997	24.4	6.0151	14.2
5.714	2			5.7359	5.1
5.4451	6.7			5.568	3.9
5.1587	4.1			5.1845	3.2
4.8769	100	4.8874	100	4.9664	100
4.6682	11.4			4.762	5.8
4.5729	9.8	4.5635	54.3	4.6296	16.1
		4.4374	15.2	4.487	2.1
		4.0808	29.4	4.1277	33.7
4.0342	48.1			4.0773	19.9
3.8861	6.6			3.9376	3.6
3.5773	0.9			3.6044	5.6
3.4642	5.8			3.5096	3.5

**Fig. 3:** Characterizing lipid components of mouse liver HLD. Thin-layer chromatography of HiF diet induced NAFLD livers. Lecithin, cholesterol, and cholesterol oleate were used as TLC standards as they were the most likely HLD components. Control liver had no TLC activity in this range while both mouse and patient NAFLD samples showed TLC reactions in cholesterol, and cholesterol oleate ranges

### Liquid crystals in HiF diet induced NAFLD animals are destroyed by conventional histological treatment

Although hepatic lipid accumulation was detected as optically active birefringent structures in all HiF diet specimens, liquid crystal (LC) is the in vivo form of hepatic lipid droplets (HLD) accumulation. The fluidity of liquid crystals allows it to be stored in the hepatocyte cytoplasm without interfering with cellular activity. Increasing optical activity of these HLD indicates pathological increasing of lipid accumulation within hepatocytes, which leads to a larger and more molecularly stable accumulation of optically active LC. Thus, confirming and characterizing the liquid crystalline nature of birefringent structures is sufficient for identifying HLD in HiF diet induced NAFLD animals.

The article "Nonalcoholic fatty liver disease experiences accumulation of hepatic liquid crystal associated with increasing lipophagy" was published in 2020. Journal: Cell Biosci.

Hepatic lipid droplet accumulation in HiF diet induced NAFLD liver occurs as liquid crystals but not as status of liquid or crystalline lipids. NAFLD liver samples prepared as glass slide smears exhibited strong birefringent optical activity as LC-HLD Maltese crosses polarized light while control liver displayed no birefringence (Fig. 1C a, b). These Birefringent Maltese crosses correspond to the lipid droplets observed in histological images of NAFLD liver (Fig. 1D) but not found in control liver samples (data not shown). As discussed above, since these LC-HLD were only observed in cryo-section but not FEDXT prepared samples of the same livers, we hypothesized that the FEDXT treatment process necessary for conventional deparaffinization and gradient ethanol rehydration and dehydration rinses away the ethanol soluble lipids of which HLD are composed. Therefore, the vacant round and oval-shaped droplets indicated in in-set of Figure Bf are residual spaces where LC-HLD used to reside in H&E, Sirius Red and Masson’s trichrome histology slides (Fig. 1B). The minimal crystal structures found in FEDXT treated livers of HiF induced NAFLD samples are residual lipids that survived the ethanol and xylene extraction process. Thus, when the same livers are observed using cryostat section without any solvent treatment, polarized light reveals strong birefringent activity from the fully intact liquid crystals. As clinical histology is largely done on FEDXT treated samples, this hypothesis explains the lack of liquid crystals identified in patient fatty liver disease to date. The following in vitro phase transition experiments were thus conducted on cryo-sections of hepatic lipid droplets.

### HLC of HiF diet induced NAFLD animals exhibits phase transition capabilities

The unusual finding that seemingly empty vacuoles on H&E demonstrate birefringence on cryo-section was further explored and responsible particles confirmed to be LC-HLDs. By successfully completed phase transitions between two of three physical states, isotropic droplet, liquid crystal HLC, and complete crystal, HLDs were confirmed to be liquid crystalline in nature. All phase transitions exhibited were conducted on both cryo-section tissues and smear specimens obtained from HiF diet induced NAFLD mice. All three physical states were detectable when the necessary phase transition conditions were met (Table 2). HiF diet induced liver smear specimens were able to transition from LC-HLD to anisotropic crystal (Ph_ani-LC→ani-CRYST_ transition) when the temperature was lowered to 0 °C. These crystal structures then retained their structure when restored to room temperature (Figs. 3B a, 4A①). When LC-HLDs were heated to 39 °C, the birefringence of Maltese crosses vanished into non-birefringent hepatic isotropic droplets (Ph_ani-LC→iso-HLD_ transition) (Figs. 4A②, 5a–h). Crystalline HLDs could also be restored to isotropic lipid droplets (Ph_ani-CRYST→iso-HLD_ transition) when the temperature is increased to 42 °C (Fig. 4A③, B a–h). Isotropic lipid droplets can be transitioned into two forms depending on the speed of temperature change during the phase transition process. Decreasing temperature quickly (fast-cooling) leads isotropic lipid droplets to resume the Maltese Crosses birefringence of anisotropic droplets (Ph_iso-HLD→ani-LC_ transition) (Figs. 4A④, B i–p and 5i–p). However when temperature is decreased slowly (slow-cooling), isotropic droplets adopt birefringent crystal structures (Ph_iso-HLD→ani-CRYST_ transition) (Fig. 4A⑤).

The article "Nonalcoholic fatty liver disease experiences accumulation of hepatic liquid crystal associated with increasing lipophagy" was published in 2020. Journal: Cell Biosci.

**Table 2:** Phase transitions of crystal structure and isotropic NAFLD HLC

Optical activity	Crystal birefringence initially disappears	Crystals transit into isotropic HLDs	Crystal birefringence initially resumes	Isotropic HLDs transit back to crystals
mV	1.67	1.52	1.41	1.36
T (°C)	40.2	42.0	36.5	35.5

**Fig. 4:** Phase transitional properties of crystalline hepatic lipid droplets (HLDs) obtained from HiF diet induced NAFLD livers. **A** Phase transitions between anisotropic liquid crystal (ani-LC), anisotropic crystal (ani-CRSYT), and isotropic lipid droplet (iso-HLD) were labeled with ① to ⑤ with arrows indicating direction of phase transition. **B** Recording of transition from anisotropic crystal to isotropic hepatic lipid droplet with temperature increase to 42 °C are shown in panels a to h and return to anisotropic liquid crystal with return to room temperature are shown in panels i to p. The difference in optical activity of crystalline, anisotropic droplet, and liquid crystal phases in a single view are shown in panels q, r, and s. Panel q shows the birefringence density of a crystal HLD, panel r shows the lack of birefringence of an anisotropic HLD, and panel s shows the birefringence density of a liquid crystal HLD. Panel t shows the typical birefringence shape of a crystalline HLD while panel u shows the post transition liquid crystal HLD demonstrating signature Maltese cross birefringence. Scale bars are 40 μm in panels a to m; 25 μm in panels t and u

**Fig. 5:** Birefringence recovery by liquid crystal hepatic lipid droplets after an isotropic lipid droplet transition. Images of HiF diet induced NAFLD HLD phase transition from liquid crystal to isotropic lipid droplet are shown in **a**–**h**. The resumption of birefringence as HLD regain liquid crystalline form is shown in **i**–**p**. Optical activity of this process is quantified in **q**, **r** and **t**. **q** Birefringence density of the initial liquid crystal, **r** the lack of birefringence in anisotropic hepatic lipid droplets, and **s** birefringence density of recovered liquid crystal HLDs. **t**, **u** Demonstrate that both the initial and recovered liquid crystalline HLDs exhibit signature Maltese cross birefringence. Scale bars are 40 μm in **a**–**p**; 25 μm in **t** and **u**

Time lapse recordings were used to document the phase transitional properties of hepatic lipid droplets from HiF diet induced NAFLD mice. Birefringent crystal structures from the liver of NAFLD mice were freshly harvested at the end of a 25 week HiF diet and immediately cryo-sectioned, mounted with PBS, and their phase transitions processes recorded as pre previously published protocols [23, 26]. To retain maximum HLD content, samples used for phase transition studies were not treated with solvents (i.e. formaldehyde, ethanol, methanol, and xylene) and recordings were carried out in 30% glycerol PBS between glass slides and coverslips.

The article "Nonalcoholic fatty liver disease experiences accumulation of hepatic liquid crystal associated with increasing lipophagy" was published in 2020. Journal: Cell Biosci.

Fresh sections of HiF diet induced NAFLD livers obtained using cryo-stat showed birefringent crystal structures under crossed polarization lights (Fig. 4B a and t) and their optical activities quantified in Fig. 4B q. When specimen temperature was increased to 42 °C, these birefringent crystal structures disappeared as the Ph_ani-CRYST→iso-HLD_ phase transition was triggered (Fig. 4B a–h) and the lack of optical activity quantified in Fig. 4B r. When these heat induced isotropic specimens were then fast-cooled, they resumed the typical optical activity of liquid crystals immediately (Fig. 4B i–p). These post Ph_iso-HLD→ani-LC_ phase transition birefringent Maltese crosses are shown in Fig. 4B p and u and quantified in Fig. 3B s. When the same heat induced isotropic specimens were slow-cooled, the isotropic hepatic lipid droplets assumed crystal structures typical of the Ph_iso-HLD→ani-CRYST_ phase transition (not shown). The ability of these LC-HLDs to assume crystalline form in slow-cooling conditions explains the crystalline structures found on our previously described X-ray diffraction studies. The phase transitions documented above hold true in both cryo-sections and smear preparations of HiF diet induced NAFLD livers. The ability of HLDs in HiF diet induced NAFLD mice to complete the above phase transitions confirm them to be liquid crystalline in nature.

### HLD from HiF diet induced NAFLD exhibit liquid crystalline fluidity

Fluidity and optic activity are the main properties of liquid crystals that distinguish them from pure crystal or liquid states. Thus, to supplement the described birefringence transitions between liquid crystal lipid droplet, isotropic lipid droplet and crystal HLD, here we describe the fluidity of these NAFLD LC-HLD. The following studies were conducted using the classic pressure-and-release procedure (P&R).

All specimens were prepared using the previously described fresh cryo-section method to retain maximum HLD content. These samples were first heated to 42 °C then fast-cooled immediately to 10 °C for 30 s before being allowed to resume room temperature (Fig. 5a–p). This Ph_iso-HLD→ani-LC_ process grants the greatest yield of liquid crystalline HLDs (Fig. 5q, s and t) by optical activty. These LC-HLD samples were then placed between polarized prisms (polarizer and analyzer) for P&R studies. Prior to pressure application, LC-HLD appeared as round droplets of various sizes. Under polarized light, all droplets retained the characteristic four equally sized quadrants of birefringence known as liquid crystal Maltese crosses. Once pressure was applied, these NAFLD LC-HLD demonstrated their fluidity by adapting a dramatic range of pressure induced shape changes.

Factual to liquid crystal states, when pressure was removed these LC-HLDs were also able to regain their original shape and classic Maltese cross birefringence. Directly after pressure release, fusion between individual LC-HLDs are seen as the particles reconsolidate. Double fusion events between LC-HLD occurs as sequential events (Fig. 6A) with one fusion (Fig. 6A j–r) occurring after the completion of a previous fusion (Fig. 6A a–i). These multiple fusions dramatically change the volume of a single LC-HLD while maintaining total volume of the all involved particles (Fig. 6A s and t). Multiple extrusions were also documented after P&R application. Double extrusions occur sequentially with one large LC-HLD extruding two individual droplets, one (Fig. 6B g–j) after another (Fig. 6B a–e). Unsuccessful extrusion with incompletely fusion of the droplets are also seen as in-and-out oscillation movements between a group of LC-HLDs (Fig. 6C a–i). These LC-HLDs are confirmed as one interacting group by tracing the stable volume of the whole complex (Fig. 6C m). These fluidity behaviors typical of LC-HLDs on P&R procedure confirm their liquid crystalline nature.

The article "Nonalcoholic fatty liver disease experiences accumulation of hepatic liquid crystal associated with increasing lipophagy" was published in 2020. Journal: Cell Biosci.

**Fig. 6:** Hepatic lipid droplets from HiF diet induced NAFLD livers demonstrate liquid crystal fluidity. **A** Sequential fusion of LC-HLDs were documented during the pressure-and-release (P&R) protocol. The first fusion shown in panels a to i is composed of two stages. In stage 1, a row of smaller LC-HLDs (S2 and S4 in panel s diagram) is lined up next to a large LC-HLD (S1 in panel s diagram) (panels a to d). During stage 2, the first small S2 LC-HLD fuses with the larger S1 LC-HLD (1st fusion of LC-HLD S2 to S1; panels e–i). A second fusion of a smaller S3 LC-HLD then follows the same mechanism (panels j to r). In this process, S3 LC-HLD first lines up with LC-HLDs S1 and S4 (panels j to k) before beginning the fusion process (panels l to r). The sequential fusion process is diagramed in panel s and the consequent volume changes confirming the LC-HLD merge are documented in panel t. **B** Sequential extrusions of LC-HLDs from a larger LC-HLD were also documented during the P&R protocol. The first extrusion is shown in panels a to d. Once the first LC-HLD droplet is fully extruded (panels e to j), a second extrusion begins (panels g to i) and successfully separates in panel j. The two sequential extrusions are diagramed in panel k and volume alternations during extrusion of LC-HLD S1 and S2 are documented in panel l. **C** An unsuccessful extrusion is recorded as in-and-out oscillations of a large, oblong LC-HLD. First a smaller LC-HLD (S2) is seen merging into a larger LC-HLD (S1) completely (panels a to g), before a new smaller LC-HLD (S3) forms and attempts to separate from the larger LC-HLD S1 (panel c to f). During this unsuccessful extrusion, the S3 merges back with the larger S1 (panel h to i) while the location S2 previously occupied begins to exhibit the formation of a new LC-HLD (S2*) (panel h to l). This in-and-out oscillation movement is diagramed in panel m, and volume alternations of LC-HLD S1, S2 and S3 are documented in panel n. Volume of individual and fusional LC-HLD sphere(s) were calculated using $V_{sph} = \left( {\frac{\pi }{3}} \right)\left[ {h_{1}^{2} \left( {3r_{1} - h_{1} } \right) + h_{2}^{2} \left( {3r_{2} - h_{2} } \right)} \right]$ (h, spherical cap; r, spherical radius)

### Crystal crystals and phase transition in early patient fatty-liver disease

As characterized above, livers of mice with HiF diet induced NAFLD exhibit liquid crystal identifying phase transition and fluidity characteristic. Confirmation of these physical properties in patient liver disease represents a potential novel method for diagnosing and characterizing patient NAFLD and may serve as a parameter for studying progression to severe symptomatic steatohepatitis, fibrosis, and cirrhosis. To adapt our animal model findings to clinical use, we conducted liquid crystal phase transition and fluidity tests on patient fatty liver disease specimens. In patient NAFLD specimens, we identified hepatic lipid droplets exhibiting Maltese-cross birefringent droplets with inner-non-activity (Fig. 7A a), full Maltese-cross birefringent activity (Fig. 7A b), and crystalline birefringence (Fig. 7A c).

The article "Nonalcoholic fatty liver disease experiences accumulation of hepatic liquid crystal associated with increasing lipophagy" was published in 2020. Journal: Cell Biosci.

**Fig. 7:** Comparisons between optical properties of LD-HLD from NAFLD patients and HiF diet induced NAFLD mice. **A** LC-HLDs from patients (pLC-HLDs) display three types of birefringence, inner-non activity (INA) Maltese-cross birefringence, full birefringent activity (FBA) Maltese-cross birefringence, and crystalline birefringence (panel Aa, Ab and Ac). Optical activity of pLC-INA and pLC-FBA lipid droplets are similar to optical properties of INA and FBA LC-HLD from HiF diet induced NAFLD mouse livers (panel f and g). **B** Plate rotation demonstrates that the pattern of optical activity in pLC-INA is independent from rotation angle (α) ranging from 0° to 360° (panel a–i). Strong birefringence remains on the cortical edge of pLC-HLDs (arrows) regardless of the changing angle of polarized light (top in panel a, c, e, g and i, and bottom in panel b, d, f and h), indicating that optical activity is restricted to the cortex of a spherical droplet

Optic activity in inner-non-activity (INA) Maltese-crosses is restricted to the cortex of hepatics lipid droplets while the center of the droplet remains dark (Fig. 7A lower middle column). This finding indicates that in early fatty liver disease lipid molecules are ordered on the outer surface of the droplet, but remains relatively chaotic within the HLD core. Although most droplets are in the described INA Maltese-cross form, some droplets do exhibit full birefringent activity (FBA) Maltese-cross birefringence (Fig. 7A lower right column). These FBA Maltese-crosses are optically identical to the Maltese-crosses observed in the LC-HLDs of our NAFLD mice (Fig. 7A lower left column). A possible link between INA Maltese-cross birefringence and FBA Maltese-cross birefringence is indicated by phase transitional properties previously shown in NAFLD mouse LC-HLD. During the Ph_iso-HLD→ani-LC_ phase transition, INA Maltese-crosses lose birefringence in the cortical layer and become isotropic HLD. Although these isotropic INA HLD Maltese-crosses still regain optical activity after fast-cooled in the Ph_iso-HLD→ani-LC_ phase transition, these post phase transition HLDs also retain the lack of central optical activity as INA Maltese-crosses (not shown). This indicates that in early fatty liver specimens, the cortex molecule order is unadulterated by transitions but the core of HLDs remain unable to order themselves despite a transitional period in the higher entropy droplet form. This central defect is confirmed to be restricted to the midpoint by observing the samples at from the full 360° range (Fig. 7B). Aside from the focal loss of optical activity, these patient fatty liver disease HLDs retain the fluidity and phase transitional properties of liquid crystals (data not shown).

The article "Nonalcoholic fatty liver disease experiences accumulation of hepatic liquid crystal associated with increasing lipophagy" was published in 2020. Journal: Cell Biosci.

Our data demonstrate that the Ph_iso-HLD→ani-LC_ phase transition occurs in both the liquid crystal hepatic lipid droplets of HiF diet induced NAFLD animals and NAFLD patients. In both the NAFLD model and patient, decreasing temperature transitions LC-HLDs from isotropic droplets to the liquid crystal phase. In liquid crystal physics, phase transition occurs with increasing concentrations of component parts. In the case of HLDs, the build-up of lipids such as cholesterol oleate within the hepatocyte. The tri-lipid cholester-phospholipid-cholesterol system is widely recognized as the system of lipid storage representative of biological system [27]. Thus, we hypothesize that the unremittent over consumption of nutrients leading to fat storage would eventually trigger the INA Maltese-cross birefringent HLDs to develop into FBA Maltese-cross birefringent HLD. With further over nutrition, these FBA Maltese-cross HLDs would eventually reach a concentration of lipids that would trigger the Ph_ani-LC→ani-CRYST_ phase transition. Since crystal are much less adaptable to the fluidity of cellular workings, they damage hepatocytes and lead to clinically detectable liver fibrosis and cirrhosis.

### Autophagy is downregulated in NAFLD hepatocytes with excess LC-HLD accumulation

As demonstrated by our high fat diet induced NAFLD mouse model and clinical progression, NAFLD is a disease associated with metabolic syndrome. In the setting of metabolic syndrome, lipophagy regulates intracellular lipid stores in an extracellular nutrition sensitive manner. As lipophagy functions via lysosomal degradation of autophagocytosed LD triglycerides, is an efficient method of removing extra cellular lipid over-accumulation [28, 29]. To assess the involvement of autophagy in LC-HLD accumulation, we compared the expression and distribution of autophagy marker microtubule-associated protein light chain 3 A (MAP1LC3A) in the livers of normal diet control mice, HiF diet induced NAFLD mice, and patient NAFLD. In control mouse livers, MAP1LC3A is highly and homogenously expressed in hepatocytes with slightly less distribution along the central veins. This even distribution of MAP1LC3A corresponds with the even but sparse distribution of LC-HLD in these samples (Fig. 8A top row) with no birefringence activity (Fig. 8A d). In HiF diet induced NAFLD mouse livers, MAP1LC3A expression all but vanished with very faint expression accompanying areas of unusually large LC-HLDs accumulations (Fig. 8A middle row) with massive birefringent LC-HLDs (Fig. 8A i). This reduced MAP1LC3A expression is reflected in patient NAFLD livers, where patient samples exhibit dramatically low expression of MAP1LC3A (Fig. 8A bottom row) with a few birefringent LC-HLDs (Fig. 8A n). The reduced expression of MAP1LC3A in mouse NAFLD samples was statistically lower than that of the normal liver samples (Fig. 8B, ***p < 0.0001, *p *= 0.000005). This lower MAP1LC3A expression was seen throughout the liver without bias between distance to the liver capsule or central vein (Fig. 7C). To confirm the involvement of autophagy in LD-HLD formation, Beclin-1 expression was analyzed via western blot and showed the same reduction in mouse (Fig. 8D, **p < 0.01, *p* = 0.0025). Both expression of MAP1LC3A and Beclin 1 in patient is exhibited much lower in immunostaining (Fig. 8A m–q, B) and Western blotting (Fig. 8D) but not vanished indicating possible tendency of lipophagy in development of fatty liver disease. No detectable difference were found in histological images between normal livers of human and mouse in publications up to date.

The article "Nonalcoholic fatty liver disease experiences accumulation of hepatic liquid crystal associated with increasing lipophagy" was published in 2020. Journal: Cell Biosci.

**Fig. 8:** Expression of MAP1LC3A implicates lipophagy in HiF diet induced NAFLD. **A** Control mouse hepatocytes exhibit strong MAP1LC3A activity throughout the liver with a slightly muted expression near vasculature and bile ducts (panel a to c). These control livers exhibit no optical activity under polarization microscopy (panel d) and contain no large vacuoles indicating hepatic lipid droplet accumulation (panel e). MAP1LC3A expression is reduced in HiF diet induced NAFLD mouse livers (panel f to h). In these livers, massive Maltese cross birefringent LC-HLDs (panel i) are seen in locations corresponding to empty vacuoles found on H&E stain (panel j). MAP1LC3A expression was not as dramatically reduced in patient NAFLD and retained some expression near the bile network (panels k to m). These patient NAFLD samples were also optically active, with both INA and FBA (panel n) birefringent particles occupying space seen as empty vacuoles on H&E (panel o). Bars are 100 μm in length. Bars in panel **A** are all 100 μm in length. **B** Quantified comparison of MAP1LC3A expression via immunostaining is shown. Mouse NAFLD samples showed significantly reduced MAP1LC3A expression (***p < 0.0001). **C** ImageJ analysis of MAP1LC3A distribution in livers organized as proximity to the central vein (CV) or lobule boundary (LD), generated with ImageJ interactive 3D surface plot. Top row shows MAP1LC3A expression in a control liver, middle row shows MAP1LC3A expression in a HiF diet induced NAFLD mouse liver, and bottom row shows MAP1LC3A expression in a patient NAFLD liver. **D** Western expression of Beclin 1, another autophagy marker, was used as secondary confirmation of autophagy deactivation. Both Beclin 1 expression is significantly down-regulated in the mouse model (mNAFLD) livers in comparison to control liver and normalized to β-actin internal control (**p < 0.01). All statistical analyses were conducted using triplicate data

These observations suggest that lipophagy is involved in the formation of LC-HLD. In normal physiological conditions, expression of MAP1LC3A in hepatocytes suggests autophagy is key in maintaining lipid homeostasis via LC-HLD storage. However in pathological accumulation of LC-HLD, MAP1LC3A signaling is down regulated except in areas with greater than normal LC-HLD accumulation. This finding concurs with previous findings that impaired lipophagy can lead to excessive intracellular lipid accumulation and leads to two theories of cause and effect. One implies impaired lipophagy as the cause of LC-HLD accumulation, while the second addresses the heretofore unknown mechanism through which intracellular lipid levels regulate lipophagy [30]. As demonstrated by their recoveries from deformations during fluidity tests, fully liquid crystalline HLD structures have great tensile strength. The strength of these non-covalent bonds between lipid molecules may provide resistance to and down regulation of effective lipophagy, thereby offering an alternative explanation for the lack of MAP1LC3A expression in NAFLD samples.

The article "Nonalcoholic fatty liver disease experiences accumulation of hepatic liquid crystal associated with increasing lipophagy" was published in 2020. Journal: Cell Biosci.

## Discussion

Over-nutrition has been recognized as the direct cause of Non-alcoholic fatty liver disease and the associated pathological hepatocyte lipid deposition. Although NAFLD is initially asymptomatic, disease progression can lead to the development of sever liver diseases such as steatosis, steatohepatitis, fibrosis, cirrhosis, and hepatocellular carcinoma [2, 5–7]. The progression of NAFLD before it begins to affect liver function is notoriously difficult to monitor. The liquid crystal properties of HLD in our HiF diet induced NAFLD mice may be a first step towards a method of monitoring the disease and projecting prognosis. Phase transition and fluidity tests on HLDS would reveal the degree of liquid crystalline organization HLDs have achieved, and thus the progression into the more damaging crystalline form once a critical lipid concentration is reached.

Although liquid crystals are not usually found in normal adult tissues and organs, they are prevalent during the developmental process. From embryonic development to postnatal day 14 in the chicken, liquid crystalline structures can be observed in more than twenty organs and tissues [24]. A tubular network of liquid crystal was also recently identified during in vitro differentiation of patient stems into embryoid bodies. This complex liquid crystal network formed during the gastrulation-like tissue and is reminiscent of a primitive vascular architecture charged with distributing resources to all the components of the differentiating embryoid body [29]. Similar to intrinsic signaling pathways being mistakenly reactivated in disease, we theorize that liquid crystalline structures are a previously undefined but important primordial system that is commonly reactivated in diseased states. For example, Anderson–Fabry disease, a disease of glycophospholipid or glycosphingolipid (GL) (globotriaosylceramide and galabiosylceramide) accumulation in the endothelial and smooth muscles cells of blood vessels also results in intracellular liquid crystalline particles [31–36]. This common occurrence of liquid crystalline structures in highly disparate diseases hints at an innate importance of liquid crystals to cellular function that needs to be further investigated as in the case of NAFLD.

There are two main reasons liquid crystals have thus so far been overlooked in human pathology. First, traditional histological examination of patient livers paraffin embed the samples and treat the resultant slides to a variety of solvents. The consequent deparaffinization, rehydration, and dehydration process using xylene and ethanol then proceeds to strip away the hepatic lipid droplets, leaving behind only the empty vacuoles stereotypical of hepatosteatosis. In support of this reasoning, cryo-section samples undergoing H&E, Sirius Red, and Masson’s trichrome staining contained only empty vacuoles under polarized light while sequential sections without such treatment exhibited birefringent hepatic lipid droplets within these seemingly vacant spaces [16, 17]. Second, the temperatures sensitive nature of liquid crystals makes them difficult to identify directly after cryo-section. When the NAFLD tissues are sliced in optimal cutting temperature compound, the low temperature causes LC-HLDs to undergo the Ph_ani-LC→ani-CRSYT_ phase transition and remain crystalline. Thus, immediate observation without treatment will only perceive crystal structures under polarized light. Because of both these circumstances, the current clinical standard-of-care for patient biopsies and traditional histological analysis would only provide a look at cellular structure but not the observations of liquid crystalline HLDs [15, 16].

The article "Nonalcoholic fatty liver disease experiences accumulation of hepatic liquid crystal associated with increasing lipophagy" was published in 2020. Journal: Cell Biosci.

New diagnostics procedures such as high intensity focused ultrasound (HIFU) and magnetic resonance elastography (MRE) have recently been developed as powerful noninvasive techniques to evaluate severity of liver damage in NAFLD and nonalcoholic steatohepatitis [37–39]. Although these techniques are efficient at determining whether patients with end-stage liver disease can be managed with stricter weight management or require transplantation, they are of limited effectiveness in early stage NAFLD. Because early intervention in HAFLD is crucial for determining treatment recommendations and reducing disease progression, another method of assessing this group of patients is necessary. Here we report the liquid crystal biophysical property of HLDs as a potential method for assessing the existence of early fatty liver disease in metabolic syndrome patients. At minimum, the fluidity and phase transition assays used to confirm liquid crystal status can be conducted on a small portion of a biopsy sample. Thereby providing valuable information with without damaging the current clinical flow for this gold standard clinical test [40, 41]. Indeed the Ph_ani-CRYST→iso-HLD_ and Ph_ani-LC→iso-HLD_ phase transition temperatures may provide valuable information as cholesterol levels have been known to affect the lattice behavior of liquid crystal in phase transition and thus alter transitional temperatures [39–41].

Here we describe the degree of birefringence advancing from the cortex of LC-HLD as a possible indication for level of HLD lipid saturation. In order to function smoothly, all cells must sequester important hydrophobic components from its largely water-soluble environment. Hepatocyte accomplishes this task by sequestering its lipids as hepatic lipid droplets with the hydrophilic head of amphiphilic lipid molecules facing the surrounding cytoplasm and hydrophobic portions projecting internally. As the concentration of amphiphilic lipid molecules increases, the non-covalent forces between amphiphilic molecules overwhelms the inherent inclination towards a high entropy, chaotic core to form internal lipids organize into alternating hydrophilic and hydrophobic layers. Because of this tight orientation, these hepatic lipid droplets gain liquid crystal birefringence in polarized light and retain the fluidity of liquid crystals. Further accumulation of lipids in hepatocytes past this point leads to over-saturation of the system and transition of liquid crystal HLD into crystalline HLD, which are rigid and likely to cause hepatocellular damage. Thus, systematic examination of patient samples under polarized light might provide key evidence on the severity of NAFLD. Such information would be invaluable in providing prognostic information on the progression of the disease into the more severe forms of disease. With such information in hand, more aggressive treatments can be initiated to prevent patients from developing steatohepatitis, fibrosis, and cirrhosis.

The article "Nonalcoholic fatty liver disease experiences accumulation of hepatic liquid crystal associated with increasing lipophagy" was published in 2020. Journal: Cell Biosci.

In lipid-rich conditions, the apo-CIII protein is thought to function as a promotor of hepatocellular triglyceride uptake and triglyceride-rich VLDL assembly [42–44]. We hypothesize that during HiF diet over-nutrition, apo-CIII are distributed on the surface of liquid crystal HLD as they are on the surface of VLDL particles. From these surface locations, apo-CIII could collect and assimilates cholesterol and cholesterol derivatives into the HLD on which it resides. This gives the gene a critical role in lipid accumulation within LC-HLDs. And supports the strong association of promoter region polymorphism in *apolipoprotein C3* (*APOC3*) (rs2854117 [− 482C>T] and rs2854116 [− 455T > C]) found to be strongly associated with NAFLD and its associated diseases, hypertriglyceridemia, metabolic syndrome, and coronary artery disease [45–48]. Thus, polymorphisms in the *APOC3* gene resulting in greater than normal incorporation of cholesteric lipids into LC-HLDs would put the individual at greater risk of over saturating the HLDs liquid crystal buffering system and transitioning the HLD into its damaging crystalline form.

In addition to the *APOC3* polymorphism described above, variations of *PNPLA3* and *TM6SF2* have also been linked to severe hepatic steatosis. Although the results are inconclusive, these genes are thought to contribute the disease by affecting hepatic triglyceride metabolism [11, 12]. Our previous study showing that liver-specific overexpression of *NG37* induced fatty liver disease in a high fat diet dependent manner also put this new member of the von Willebrand A (vWA) super family on the map of metabolic diseases [15]. These high fat diet liver-specific overexpression of *NG37* mice developed rapid hepatocellular liquid crystalline lipid accumulation that was greater than both high fat-diet wild type litter mates and normal diet *NG37* mutant mice. In addition to liver enlargement and steatosis, these mice also developed cardiac arrhythmias commonly seen in NAFLD patients. This evidence clearly points at the importance of *NG37* in hepatocellular lipid metabolism and NAFLD. Further studies are currently investigating the links between metabolism syndromes, cardiac function, and *NG37*. In this study, we found that MAP1LC3A a marker of lipophagy, lipid specific autophagy, is dramatically down-regulated in over-nutrition induced NAFLD liquid crystal hepatic lipid droplet accumulation. As exercise can improve lipid over accumulation by increasing lipophagy [49, 50], the next step is to investigate whether exercise can reactivate MAP1LC3A associated autophagy. Understanding the relationship between liquid crystal hepatic lipid droplets and the MAP1LC3A autophagy could provide a unique prospective towards understanding, preventing, and treating NAFLD.

The article "Nonalcoholic fatty liver disease experiences accumulation of hepatic liquid crystal associated with increasing lipophagy" was published in 2020. Journal: Cell Biosci.

## Conclusions

Characterization of liquid crystal hepatic lipid droplets in mouse and patient NAFLD samples is a novel mechanism based on phase transition for evaluating the level of hepatic steatosis. Our discovery of hepatic lipid droplets with no core optical birefringence hints at the role cholesterol saturation plays in liquid crystal hepatic lipid droplet formation. By the laws of physics, as concentration of amphiphilic molecules increase it become energetically sensible to shift from a chaotic core of amphiphilic molecules protected by a layer of external facing hydrophilic molecules into a solid sphere of alternating hydrophilic and hydrophobic layers. This finding indicates that studying the degree of birefringence in patient hepatic lipid droplets may reveal disease severity long before patients become symptomatic. The greater the cholesterol content, the more thorough the droplet birefringence, and the closer a droplet comes to reaching full lipid saturation, at which point the liquid crystal droplet becomes crystalline. These less malleable droplets then cause hepatic damage, leading to steatohepatitis, fibrosis, and cirrhosis. Thus, identifying the degree of hepatic lipid droplet birefringence could be a novel diagnostic for NAFLD patients.

## Data Availability

The data set supporting the conclusions of this article are included within the article.

## Abbreviations

ani-CRSYT: Anisotropic crystal
ani-LC: Anisotropic liquid crystal
APOC3: Apolipoprotein C3
FBA: Full birefringent activity
FEDXT: Formaldehyde fixation, ethanol gradient dehydration, and xylene for transparent
GL: Glycophospholipid or glycosphingolipid
H&E: Hematoxylin and Eosin
HiF: High fat
HIFU: High intensity focused ultrasound
HLD: Hepatic lipid droplets
INA: Inner optical activity
iso-HLD: Isotropic lipid droplet
LC-HLD: Liquid crystal hepatic lipid droplets
LD: Lipid droplets
MAP1LC3A: Microtubule-associated protein light chain 3 A
MRE: Magnetic resonance elastography
NAFLD: Non-alcoholic fatty liver disease
NASH: Nonalcoholic steatohepatitis
P&R: Pressure-and-release procedure
PNPLA3: Patatin like phospholipase domain containing 3
TLC: Thin-layer chromatography
TM6SF2: Transmembrane 6 superfamily 2
vWA: von Willebrand A
XRD: X-ray diffraction

The article "Nonalcoholic fatty liver disease experiences accumulation of hepatic liquid crystal associated with increasing lipophagy" was published in 2020. Journal: Cell Biosci.

## References

[1] Shaker M, Tabbaa A, Albeldawi M, Alkhouri N (2014). Liver transplantation for nonalcoholic fatty liver disease: new challenges and new opportunities. World J Gastroenterol.

[2] Rinella ME (2015). Nonalcoholic fatty liver disease: a systematic review. JAMA.

[3] Yen CH, Wang KT, Lee PY, Liu CC, Hsieh YC, Kuo JY (2017). Gender-differences in the associations between circulating creatine kinase, blood pressure, body mass and non-alcoholic fatty liver disease in asymptomatic asians. PLoS One.

[4] Zhang Q, Wong CKH, Kung K, Chan JCY, Sy BTW, Lam M (2017). Development and validation study of a non-alcoholic fatty liver disease risk scoring model among adults in China. Fam Pract.

[5] Moran JR, Ghishan FK, Halter SA, Greene HL (1983). Steatohepatitis in obese children: a cause of chronic liver dysfunction. Am J Gastroenterol.

[6] Chalasani N, Younossi Z, Lavine JE, Diehl AM, Brunt EM, Cusi K (2012). The diagnosis and management of non-alcoholic fatty liver disease: practice guideline by the American Association for the Study of Liver Diseases, American College of Gastroenterology, and the American Gastroenterological Association. Hepatology.

[7] Clark JM, Diehl AM (2003). Nonalcoholic fatty liver disease: an underrecognized cause of cryptogenic cirrhosis. JAMA.

[8] Wang F-S, Fan J-G, Zhang Z, Gao B, Wang H-Y (2014). The global burden of liver disease: the major impact of China. Hepatology.

[9] Wong VW-S, Chan W-K, Chitturi S, Chawla Y, Dan YY, Duseja A (2018). The Asia-Pacific working party on nonalcoholic fatty liver disease guidelines 2017 part 1: definition, risk factors and assessment. J Gastroenterol Hepatol.

[10] Anderson EL, Howe LD, Jones HE, Higgins JPT, Lawlor DA, Fraser A (2015). The prevalence of non-alcoholic fatty liver disease in children and adolescents: a systematic review and meta-analysis. PLoS One.

[11] Romeo S, Kozlitina J, Xing C, Pertsemlidis A, Cox D, Pennacchio LA (2008). Genetic variation in PNPLA3 confers susceptibility to nonalcoholic fatty liver disease. Nat Genet.

[12] Kozlitina J, Smagris E, Stender S, Nordestgaard BG, Zhou HH, Tybjaerg-Hansen A (2014). Exome-wide association study identifies a TM6SF2 variant that confers susceptibility to nonalcoholic fatty liver disease. Nat Genet.

The article "Nonalcoholic fatty liver disease experiences accumulation of hepatic liquid crystal associated with increasing lipophagy" was published in 2020. Journal: Cell Biosci.

[13] Petersen KF, Dufour S, Hariri A, Nelson-Williams C, Foo JN, Zhang XM (2010). Apolipoprotein C3 gene variants in nonalcoholic fatty liver disease. N Engl J Med.

[14] Zhang H, Chen L, Xin Y, Lou Y, Yang L, Xuan S (2014). Apolipoprotein C3 gene polymorphisms are not a risk factor for developing non-alcoholic fatty liver disease: a meta-analysis. Hepatitis Mon.

[15] Zhou X, Xu M, Wang L, Mu Y, Feng R, Dong Z (2016). Liver-specific NG37 overexpression leads to diet-dependent fatty liver disease accompanied by cardiac dysfunction. Genes Nutr.

[16] Ioannou GN, Haigh WG, Thorning D, Savard C (2013). Hepatic cholesterol crystals and crown-like structures distinguish NASH from simple steatosis. J Lipid Res.

[17] Fukuda Y, Sone T, Sakuraba H, Araki T, Ohshima T, Shibata T (2015). A novel NAD(P)H-dependent carbonyl reductase specifically expressed in the thyroidectomized chicken fatty liver: catalytic properties and crystal structure. FEBS J.

[18] Li P, Banjade S, Cheng HC, Kim S, Chen B, Guo L (2012). Phase transitions in the assembly of multivalent signalling proteins. Nature.

[19] Beutel O, Maraspini R, Pombo-Garcia K, Martin-Lemaitre C, Honigmann A (2019). Phase separation of zonula occludens proteins drives formation of tight junctions. Cell.

[20] Hofweber M, Hutten S, Bourgeois B, Spreitzer E, Niedner-Boblenz A, Schifferer M (2018). Phase separation of FUS is suppressed by its nuclear import receptor and arginine methylation. Cell.

[21] Ioannou GN, Subramanian S, Chait A, Haigh WG, Yeh MM, Farrell GC (2017). Cholesterol crystallization within hepatocyte lipid droplets and its role in murine NASH. J Lipid Res.

[22] Sundaresan S, Vijayagopal P, Mills N, Imrhan V, Prasad C (2011). A mouse model for nonalcoholic steatohepatitis. J Nutr Biochem.

[23] Ling G, Wang L, Rui F, Li Z, Wang J, Ren K (2017). Transportation of liquid crystal and CaCO_3_ vaterite crystal in chicken embryo and early postnatal development. Mol Cryst Liq Cryst.

[24] Xu M, Xu X, Sato K (2012). Liquid-crystal in embryogenesis and pathogenesis of human diseases. Embryogenesis.

[25] Xu X, Dong C, Vogel BE (2007). Hemicentins assemble on diverse epithelia in the mouse. J Histochem Cytochem.

[26] Xu XH, Xu MM, Jones OD, Chen XZ, Li YF, Yan GF (2011). Liquid crystal in lung development and chicken embryogenesis. Mol Cryst Liq Cryst.

[27] Small DM (1988). George Lyman Duff memorial lecture. Progression and regression of atherosclerotic lesions. Insights from lipid physical biochemistry. Arteriosclerosis.

[28] Goldstein JL, Brown MS (1997). The clinical investigator: bewitched, bothered, and bewildered—but still beloved. J Clin Invest.

[29] Xu MM, Jones OD, Wang L, Zhou X, Davis HG, Bryant JL (2017). Characterization of tubular liquid crystal structure in embryonic stem cell derived embryoid bodies. Cell Biosci.

The article "Nonalcoholic fatty liver disease experiences accumulation of hepatic liquid crystal associated with increasing lipophagy" was published in 2020. Journal: Cell Biosci.

[30] Liu K, Czaja MJ (2013). Regulation of lipid stores and metabolism by lipophagy. Cell Death Differ.

[31] Xu MM, Xu XH, Cao GL, Pan YX, Jones O, Bryant JL (2009). The liquid crystalline in normal renal development amplifies the comprehension for anderson-fabry disease. Mol Cryst Liq Cryst.

[32] Haimovici R, Gantz DL, Rumelt S, Freddo TF, Small DM (2001). The lipid composition of drusen, Bruch’s membrane, and sclera by hot stage polarizing light microscopy. Invest Ophthalmol Vis Sci.

[33] Lang PD, Insull W (1970). Lipid droplets in atherosclerotic fatty streaks of human aorta. J Clin Invest.

[34] Kruth HS (2001). Lipoprotein cholesterol and atherosclerosis. Curr Mol Med.

[35] Brown MS, Faust JR, Goldstein JL (1975). Role of the low density lipoprotein receptor in regulating the content of free and esterified cholesterol in human fibroblasts. J Clin Invest.

[36] Goldstein JL, Anderson RG, Brown MS (1979). Coated pits, coated vesicles, and receptor-mediated endocytosis. Nature.

[37] Ballestri S, Romagnoli D, Nascimbeni F, Francica G, Lonardo A (2015). Role of ultrasound in the diagnosis and treatment of nonalcoholic fatty liver disease and its complications. Expert Rev Gastroenterol Hepatol..

[38] Schwimmer JB, Behling C, Angeles JE, Paiz M, Durelle J, Africa J (2017). Magnetic resonance elastography measured shear stiffness as a biomarker of fibrosis in pediatric nonalcoholic fatty liver disease. Hepatology..

[39] Singh S, Muir AJ, Dieterich DT, Falck-Ytter YT (2017). American Gastroenterological Association Institute Technical Review on the Role of Elastography in Chronic Liver Diseases. Gastroenterology..

[40] Papandreou D, Rousso I, Mavromichalis I (2007). Update on non-alcoholic fatty liver disease in children. Clin Nutr..

[41] Mansoor S, Collyer E, Alkhouri N (2015). A comprehensive review of noninvasive liver fibrosis tests in pediatric nonalcoholic Fatty liver disease. Curr Gastroenterol Rep..

[42] Mendivil CO, Zheng C, Furtado J, Lel J, Sacks FM (2010). Metabolism of very-low-density lipoprotein and low-density lipoprotein containing apolipoprotein C-III and not other small apolipoproteins. Arterioscler Thromb Vasc Biol.

[43] Sundaram M, Zhong S, Bou Khalil M, Links PH, Zhao Y, Iqbal J (2010). Expression of apolipoprotein C-III in McA-RH7777 cells enhances VLDL assembly and secretion under lipid-rich conditions. J Lipid Res.

[44] Qin W, Sundaram M, Wang Y, Zhou H, Zhong S, Chang CC (2011). Missense mutation in APOC3 within the C-terminal lipid binding domain of human ApoC-III results in impaired assembly and secretion of triacylglycerol-rich very low density lipoproteins: evidence that ApoC-III plays a major role in the formation of lipid precursors within the microsomal lumen. J Biol Chem.

The article "Nonalcoholic fatty liver disease experiences accumulation of hepatic liquid crystal associated with increasing lipophagy" was published in 2020. Journal: Cell Biosci.

[45] Cao Y, Kole A, Lan L, Wang P, Hui J, Sturek M (2017). Spectral analysis assisted photoacoustic imaging for lipid composition differentiation. Photoacoustics.

[46] Miller M, Rhyne J, Chen H, Beach V, Ericson R, Luthra K (2007). APOC3 promoter polymorphisms C-482T and T-455C are associated with the metabolic syndrome. Arch Med Res.

[47] Petersen KF, Dufour S, Feng J, Befroy D, Dziura J, Dalla Man C (2006). Increased prevalence of insulin resistance and nonalcoholic fatty liver disease in Asian-Indian men. Proc Natl Acad Sci USA.

[48] Kypreos KE (2008). ABCA1 promotes the de novo biogenesis of apolipoprotein CIII-containing HDL particles in vivo and modulates the severity of apolipoprotein CIII-induced hypertriglyceridemia. Biochemistry..

[49] Flores-Toro JA, Go KL, Leeuwenburgh C, Kim JS (2016). Autophagy in the liver: cell's cannibalism and beyond. Arch Pharm Res..

[50] Chun SK, Lee S, Yang MJ, Leeuwenburgh C, Kim JS (2017). Exercise-Induced Autophagy in Fatty Liver Disease. Exerc Sport Sci Rev..

